RETRACTED

# Mechanism of Antibacterial Enhancement and Drug Resistance Based on Smart Medical Imaging on Antibiotics

**DOI:** 10.1155/2022/6103649

**Published:** 2022-03-23

**Authors:** Yanxia Xing, Xiaowen An, Boyang Wang, Guifang Chang, He Zhu, Yang Yu

**Affiliations:** College of Food Science and Project Engineering, Shandong Agriculture and Engineering University, Jinan, 250100 Shandong, China

## Abstract

With the development of antibacterial, synergistic, and drug resistance research, the requirements for the specificity of antibiotics are getting higher and higher. In the research based on the specificity of antibiotics, this article uses intelligent medical image processing methods to study the specificity of the antibacterial efficiency of nanocopper oxide and the inhibition of drug resistance. Copper oxide nanorods have the properties of surface effect, quantum size effect, volume effect, and macroscopic quantum tunneling effect. Compared with ordinary copper oxide, the nanoscale gives them special properties of electricity, optics, and catalysis. In this article, in the research based on the specificity of antibiotics, the specificity of antimicrobial efficiency and drug resistance inhibition of nanocopper oxide are studied by using smart medical information processing methods. Drug sensitivity paper tablet method is a drug sensitivity experiment to determine drug sensitivity to make accurate and effective use of drugs for treatment. Colony growth method is used to take the equivalent volume of fermentation liquid at different times to determine the content of bacteria. In this article, Staphylococcus aureus is cultivated by the drug-sensitive disk method and the colony growth method. Then, according to this type of antibiotic and bacterial group combination, Staphylococcus aureus is divided into a penicillin group, nanocopper oxide group, and cephalosporin group. 0.5 g of the corresponding antibiotic was added to each group. TMP (trimethoprim) acts as a synergist, and the ratio of TMP to antibiotic is 1 : 5. Finally, we compared the inhibitory concentration indexes of the above three groups and inferred the synergistic effect of antibiotics and the inhibitory effect of drug resistance through the specificity of the antibiotics that the antibacterial activity was further studied. The results showed that the antibacterial effect of TMP combined with nano-CuO was 38% higher than that of the penicillin group and 41% higher than that of the cephalosporin group. In addition, the combined effect of TMP and antibiotics is greater than the combined effect of TMP and antibiotics alone. From the observation of smart medical system processing, it is speculated that the reason may be that they provide each other with a suitable environment. Because of this combined effect between the TMP and the antibiotic, it can influence each other. From the results, the combined effect is 48% higher than the combined effect. Therefore, according to the results of medical imaging, the combination of antibiotics and antibacterial synergists can improve specificity and antibacterial rate.

RETRACTED

## 1. Introduction

As research into drug resistance mechanisms deepens, molecular biological studies will strongly support future drug resistance analysis. The surface polarity of liposome vesicles can improve the hydrophilicity of the drug, promote the fusion of the drug with the cell membrane of the lesion, and effectively improve the release activity and antibacterial properties of the target drug. Compared with the monomer, the antibacterial activity of nano CuO is significantly improved. It has antibacterial activity against various bacteria, especially Gram-negative bacteria, and is very valuable for further improving the antibacterial activity of antibiotics. The movement of these bacteria cannot be recognized by people under normal circumstances; some cells do not move with a flagellum but slide. Attention should be distinguished from swimming during examination. Generally, the swimming speed is high, while the sliding speed is slow. Swimming can only move in a suspension, and sliding must be attached to a solid surface. So more advanced medical imaging systems must be used. Nano-CuO fully demonstrates the antibacterial effects of antibacterial synergists against common Gram-positive and Gram-negative bacteria. The electrical properties of copper oxide nanorods make them very sensitive to the external environment, such as temperature, humidity, light, and other conditions, so the use of nanocopper oxide particle-coated sensor can greatly improve the antibacterial effect and the response speed, sensitivity, and selectivity of medical imaging; reduce resistance to conventional antibiotics; and provide effective strategies for the prevention and treatment of wound infections.

In the study of antibacterial activity, Mirabello L can improve the stability of essential oil through liposome encapsulation, thus enhancing the antibacterial activity, making plant essential oil further used as food preservatives and protectants. Although the research subjects are different from this paper, their experimental methods and experimental results are worth learning from [1]. Isakoff et al. encapsulated coconut shell extract with liposome, which not only improved the color of the extract but also enhanced the drug stability and effectively improved the antibacterial performance [2]. Inspired by this, the berberine and rhein (BER rhe) composite nanoparticles were prepared by molecular self-assembly technology (molecular self-assembly is molecules spontaneously concluded into stable, structurally determined aggregates under equilibrium conditions through noncovalent fitness. The process of spontaneously generating complex, ordered, and organized aggregate organization with specific functions through molecular self-assembly under certain conditions is termed molecular self-organization preparation), and their combined antibacterial activity was investigated [3]. In addition, nanocopper oxide of the poly(lactic acid glycolic acid) copolymer prepared by Shen et al. was used to load curcumin (cur), which solved the problems of low solubility and rapid degradation of cur [4]. Jung et al. produced a new kind of antibacterial dressing with good biocompatibility by using the image feature recognition device of the hand-held microscope. The dressing was prepared by first adding the extract of Radix isatidis to the PVP/alcohol solution and then stirring continuously at room temperature for at least 24 hours [5]. Cellulose acetate gelatin crosslinked nanofibers containing BER were similarly prepared by CHO HJ and used as wound dressings [6]. Several research cases mentioned above have promoted bacterial proliferation to some extent, but there are many deficiencies; either the research scope is too narrow, the experiment is not rigorous enough, or the significance of the research is not very great, and the antibacterial enhanced resistance mechanism of intelligent medical imaging is of great significance.

RETRACTED

In the study of Staphylococcus aureus, Xia and Wang prepared PCL-ica mixed solution and the gel-mix solution, respectively, and then extruded nanocopper oxide antibiotic mixed wire (core-shell structure) by coaxial electrospinning and mixed with protein solution to form antibacterial biomimetic periosteum [7]. Using liposomes to encapsulate antibiotics, as studied by Rong et al., not only improves the stability of antibiotics but also can bind to the porogenic toxin released by Staphylococcus aureus and perforate into the membrane [8]. Prieto-Dominguez et al. mixed Agrimonia pilosa, Rheum palmatum, Hedyotis diffusa, Polygonum cuspidatum, and other traditional Chinese medicine with silver nanoparticles to obtain corresponding drug silver nanoparticle inclusion complex. The antibacterial activity of Polygonum cuspidatum silver nanoparticle inclusion complex against Pseudomonas aeruginosa was 3000 times stronger than Polygonum cuspidatum extract, and the antibacterial activity of Geranium grandiflorum silver nanoparticle inclusion complex was also significantly improved [9]. Clayton and Ridley prepared catechol copper nanoparticles by an ultrasonic grinding method, which not only improved the stability of catechol but also realized the drug release in the pathogen site, significantly enhancing the antibacterial activity of catechol [10]. In the above studies, the combination of metal nanoparticles and effective components of traditional Chinese medicine can also produce a synergistic antibacterial effect and further improve the antibacterial activity. This encapsulation method not only failed to maximize the antibacterial activity of antibiotics but also had low safety.

RETRACTED

Based on the study of antibiotic specificity, this article uses smart medical image processing methods to study the specificity of nanocopper oxide in terms of antibacterial efficiency and drug resistance inhibition. In this paper, the susceptibility disk method and the colony growth method were used to culture Staphylococcus aureus. Then, according to the types of antibiotics combined with the flora, Staphylococcus aureus is divided into a penicillin group, nanocopper oxide group, and cephalosporin group. 0.5 g of corresponding antibiotics was added to each group. Using TMP as a synergist, the ratio of TMP to antibiotic is 1 : 5. Finally, this article compares the inhibitory concentration indexes of the above three groups and further studies the specificity of antibiotics through antibacterial activity to infer the synergistic effect of antibiotics and the inhibition of drug resistance.

## 2. Experiments and Methods of Bacteriostasis and Drug Resistance

### 2.1. Research Content

The andrographolide (andrographolide is an organic substance, white square prism or flake crystal. The main active ingredient of the natural plant Andrographis paniculata has the functions of dispelling heat and detoxification, reducing inflammation, and relieving pain and has special effects on bacterial and viral upper respiratory tract infections and dysentery. It is known as a natural antibiotic drug) used in this paper is prepared by the inclusion technology-*β*-cyclodextrin inclusion compound powder and directly acts on the treatment of bacterial biological lesions of Staphylococcus aureus through a special biological delivery method. This paper is the experimental process as follows: first, determine the research content; then, prepare nanooxidation antimicrobial agent, use antibiotic synergist for proliferation; then, establish coccal resistance assessment model; and finally data analysis and conclusion. The hydrogen bonding of copper nanoparticles can effectively improve the binding ability of the nanoparticles and the surface of the bacteria so that the nanoparticles can be disintegrated on the Staphylococcus aureus membrane, and the composite nanoparticles can invade the bacteria in large quantities, thereby effectively killing the bacteria. In this paper, poly(caprolactone), polyethylene glycol (PEG), and roxithromycin (Rox) with different mass ratios were added to tetrahydrofuran and stirred at 50°C and 400 R/min for 24 h. All isolates were resistant to penicillin G but sensitive to roxithromycin, erythromycin, and streptomycin. In this article, there are seven different modes of multidrug resistance, and Staphylococcus aureus isolates show multidrug resistance. It is a nuclear medical term published in 2018, which refers to the phenomenon that malignant cancer cells are resistant to other cancer drugs with different structures and different mechanisms of action.

RETRACTED

### 2.2. Preparation of Nanocopper Oxide Antibacterial Agents

Through digital design, the porosity of drugs can be specifically controlled, and drugs with different shapes and complex internal structures can be easily printed, which can not only meet the personalized needs but also reduce the cost waste of additive manufacturing [11]. The tablets with different pores and internal structures were printed with the same material, which was a cylinder, triangular cone, and inverted triangular cone, respectively. Through comparison, it was found that different structures could produce different drug release rates to achieve different therapeutic effects [12]. First, tetracycline hydrochloride was used to prepare polymer composite membrane by a solvent casting method, and then, the antibacterial porous scaffold was prepared. The drug release in the composite membrane is linear and complete within 10 hours, while the drug stent can achieve step-by-step release after entering the body. The drug can be released rapidly in the first 10 hours and then slowly and continuously for nearly 70 hours [13]. This drug design model can be used for long-term antibacterial, which better plays the role of the stent. It can determine the proliferation effect of synergists and nanosized copper oxide antibiotics by setting physiological saline as the experimental blank control group.

The drug release kinetics and antibacterial activity are shown in Figure 1. The drug release in the 3D scaffold is more sustainable, and the antibacterial activity is more durable, which fully reflects the advantages of structure.

### 2.3. Proliferation of Antibiotic Synergist

Due to the different degradation rates of polycaprolactone and gelatin in the mixed structure of nano-CuO antibiotics, the rapid release of moxifloxacin and the long-term release of Epimedium can be achieved, respectively, which can effectively inhibit the proliferation of bacteria [14]. Nanogold, nanosilver, nanocopper, and other inorganic metal nanomaterials have significant antibacterial activity and can slow down the occurrence of bacterial resistance. This synergistic model of combining metal nanoparticles with traditional Chinese medicine can improve the antibacterial activity of traditional Chinese medicine to a certain extent, but with the continuous improvement of the number of metal nanoparticles, the problems of biological safety and price gradually become prominent, which has become the main bottleneck limiting its large-scale application [15]. For the detection of drug resistance of Staphylococcus aureus at present, the most commonly used methods for the study of drug resistance of Staphylococcus aureus are still based on phenotype test, including broth drug sensitivity test, agar plate dilution method, and disk diffusion method [16]. These traditional methods are characterized by simple operation and low cost; however, it has the disadvantages of cumbersome steps and long time-consuming [17]. With the development of genomics, many potential gene modifications that cause antibiotic resistance have been described, and the use of molecular biological methods to detect antibiotic resistance has gradually developed [18].

RETRACTED

Based on the model of Staphylococcus aureus spores, the methods of penetration and in situ signal amplification were proposed to detect antibiotic resistance genes. Compared with the traditional drug sensitivity test, the results of molecular biology techniques can be obtained more quickly and accurately by using the drug-sensitive disk method and colony growth method. However, it is uncertain that the resistance to an antibiotic may be mediated by a variety of different resistance mechanisms, and molecular methods can only be used for the resistance mechanisms previously detected and characterized; resistance to unknown or emerging antibiotics will not be detected [19]. The uniform solution was evaporated at room temperature to obtain nanocopper oxide composite material, which was melted at 95°C to prepare a new nanocopper oxide bone repair scaffold, which realized the initial sudden release bactericidal activity and later slow-release antibacterial activity and gave better play to the antibacterial effect. Moreover, peg in the scaffold improved the release rate and amount of Rox and enhanced the bioavailability, and with the increase of PEG content, the antibacterial activity of the scaffold also increased accordingly, so that the scaffold showed strong antibacterial properties [20]. This flexible adjustment of excipient dosage fully reflects the advantages of personalized pharmacy, which can facilitate the regulation of drug release activity, to improve the effectiveness and success rate of the treatment of bacterial infection. This technical advantage is not possessed by the previous several preparation technologies [21]. The advantages of the technology in the preparation of personalized antibacterial drugs are comprehensively reflected in the accurate control of antibacterial drug dosage, release rate, release time, and other parameters [22].

RETRACTED

As shown in Figure 2, the drug dosage can be “customized” according to the patient's age, course of the disease, etc. by adding and subtracting on demand; the operation is convenient; and different doses of tablets are given to different patients, to avoid the occurrence of side effects and improve the safety of the medication. It can also flexibly control the drug release rate according to the needs of the disease; accurately refer to the time effect of the drug, to achieve the best therapeutic effect; and improve the effectiveness of drug use. Through the technology to achieve long-term drug release, it can reduce the trouble of the elderly and other inconvenient people taking medicine many times and improve the convenience of drug use. The increasing drug resistance of existing antibiotics and the lack of new antibiotics being developed are threatening public health. Complex physiological and ecological environmental factors have different degrees of influence on the infection process of Staphylococcus aureus, which may disturb the absorption of drugs by fungi and even produce drug resistance, because ecological factors refer to factors that affect the morphology, physiology, and distribution of organisms in the environment. For a multicellular organism, the environment in which the whole is located is called the external environment, and the environment in which the cells that make up the organism are located is called the internal environment. The internal and external environment and life activities interact and influence each other. When the body is stimulated, the internal metabolism and external activities of the body will change accordingly [23]. Therefore, whether environmental factors promote or inhibit the occurrence of fungal drug resistance and how the mechanism of fungal drug resistance is related to environmental factors provide a certain reference for the analysis of the transmission route of drug-resistant bacteria and drug-resistant genes in the environment and the new drug resistance mechanism [24]. The control and treatment of Staphylococcus aureus infection and the development of fungal drug resistance are related to human health and environmental safety, so it is necessary to research this area [25].

RETRACTED

At present, people gradually realize that the development of microbial drug resistance will eventually threaten human health, but the discovery of new antibiotics will inevitably be accompanied by the emergence of drug resistance. The distribution and transmission path of Staphylococcus aureus are affected by human activities and the environment. However, a large number of studies are mainly focused on clinical trials or single drug research and lack of research on drug resistance and treatment mechanism of Staphylococcus aureus from the comprehensive relationship of the human soil environment. For example, the dust on the building surface and the surrounding soil in the hospital area may be the important species storehouse of human pathogenic fungi or potential human pathogenic fungi. The dust from the hospital and the soil containing bacteria in the green space may be retransmitted in the air of the hospital area through the atmosphere, ventilation equipment, or air conditioning system, thus increasing the risk of invasive fungal infection in the hospital. Therefore, it is necessary to study the relationship between humans, soil, and the environment to find a reasonable balance between the spread of fungal resistance and the control of fungal infection. The distribution, pathogenicity risk assessment, and infection route of Staphylococcus aureus were studied. The species diversity, distribution, pathogenicity risk, and possible transmission routes of Staphylococcus aureus were evaluated in specific habitats such as hospitals and zoos, and the environmental factors were comprehensively studied.

### 2.4. Evaluation Model of Coccal Resistance

Itraconazole is effective in the treatment of human dermatomycosis, and there is no clear drug resistance in patients with long-term use of itraconazole, but more than 50% of patients infected with Aspergillus fumigatus dermatosis have developed resistance to itraconazole. It should be noted that an Aspergillus fumigatus strain with azole resistance was isolated from a patient who was not infected with Aspergillus fumigatus, and this kind of Aspergillus fumigatus has high resistance to voriconazole. Antimicrobial therapy often requires the combination of a variety of drugs (such as traditional Chinese medicine and antibiotics and a variety of antibiotics) or the combination of effective components of a variety of drugs. This combination of drugs requires high preparation technology, and it is difficult for conventional technology to meet the requirements. Through the combination function (*g*) of multiple drugs, the antibacterial activity of multiple drugs can be achieved.

(1) $$\begin{array}{c} V=\frac{1}{2}{\left(t-y\right)}^{2}=\frac{1}{2}{\left[t-f\left(WX\right)\right]}^{2},\\ \Delta {WX}^{l}=-\eta \frac{\partial E}{\partial W^{l}}=\eta {\left(X^{l}\right)}^{T}\delta^{l}, \end{array}$$

where *Wx* is the posterior probability density function of reliability *E*. For the physical equipment whose test results obey binomial distribution, the uniform distribution on (0,1) can be used as the prior distribution of reliability *r* without any prior information.

(2) $$\begin{array}{c} R=\frac{e^{x}-e^{-x}}{e^{x}+e^{-x}},\\ X=\frac{x}{1+\left|x\right|}. \end{array}$$

The other is the joint distribution of sample *X* and parameter *R*.

(3) $$\begin{array}{c} R\left(v,e\right)=\left[\zeta_{1}c_{1}\left(t\right)+\zeta_{2}c_{2}\;\left(k\right)+\zeta_{3}c_{3}\left(k\right)+\zeta_{4}c_{4}\;\left(k\right)+\zeta_{5}c_{5}\left(k\right)+\zeta_{6}w_{ik}\right]. \end{array}$$

Macrophages were printed on the surface of the HA/Gel hydrogel matrix. The bone scaffold containing rifampicin, daptomycin, and macrophages was used for the prevention and treatment of biofilm infection after craniotomy. The results showed that antibiotics could be released slowly in the infected area. Although macrophages in scaffolds have no antibacterial effect, they can effectively promote the clearance of bacterial biofilms and produce a synergistic antibacterial effect with antibiotics. Further, solve the marginal distribution of sample *X*.

(4) $$\begin{array}{c} \Delta {\text{Z}}^{l3}=-{\eta \delta }^{l3}X^{l3}=\eta \left(t-y\right)f^{\prime }\left(X^{l3}W^{l3}\right)X^{l3},\\ {\text{Q}}_{ik}=\overset{n}{\underset{a}{\sum }}\tau_{1}X_{ik}+\overset{n}{\underset{b}{\sum }}\tau_{2}U\left(Y_{ik}\right)+B_{ik}. \end{array}$$

Finally, the posterior distribution of *R* is obtained.

(5) $$\begin{array}{c} c_{1}\left(t\right)\geq 0, \end{array}$$

(6) $$\begin{array}{c} \Delta R^{l3}=-{\eta \delta }^{l3}T^{l3}=\eta \left(t-y\right)f^{\prime }\left(X^{l3}W^{l3}\right)X^{l3}. \end{array}$$

Equation (6) is just the beta distribution with parameters *R* and *T*, denoted as *Q*:

(7) $$\begin{array}{c} Q_{\text{gain}}\left(Y\right)=\frac{\sigma \left(Y\right)-\text{avg}\left(\sigma \left(Y^{\prime }\right),\sigma \left(Y^{\prime }\right)\right)}{\sigma \left(Y\right)}, \end{array}$$

(8) $$\begin{array}{c} Q=\left\{\left(a_{1},b_{1}\right),\left(a_{2},b_{2}\right),\cdots ,\left(a_{n},b_{n}\right)\right\}. \end{array}$$

The information entropy 0 h (*R*) of reliability *R* can be obtained by substituting equation (7) into equation (8).

(9) $$\begin{array}{c} H{\left(R\right)}^{l3}=\left(t-y\right)f^{\prime }\left(X^{l3}W^{l3}\right),\\ A_{\lim}=f\left(x\right)=\underset{j\subset Q}{\sum }c_{j}\frac{x_{j}}{\sigma \left(X\prime_{j}\right)}-p-B,\\ N\left(d_{i},w_{j}\right)=P\left(d_{i}\right)P\left(w_{j}\left|d_{i}\right.\right),\\ P\left(w_{j}\left|d_{i}\right.\right)=\overset{K}{\underset{k=1}{\sum }}P\left(w_{j}\left|z_{k}\right.\right)P\left(z_{k}\left|d_{i}\right.\right). \end{array}$$

When introducing a certain type of historical sample FT,

(10) $$\begin{array}{c} \text{FT}=\arg\max\underset{a_{n}\in W_{K}\left(a\right)}{\sum }\left|\left(b_{n}=c_{n}\right)\right.M. \end{array}$$

The determination of super parameter *B* in beta distribution *M* can be based on the prior moment method. The process is as follows: some estimated values of reliability *R* obtained from historical data are denoted as *e*, from which the first two prior moments *T*

(11) $$\begin{array}{c} \Delta R_{i}=-\eta E^{\prime }=\eta x_{i}\left(t-y\right)f^{\prime }\left(T\right)=\eta x_{i}\delta . \end{array}$$

It not only saves the trouble of taking a variety of antibiotics but also can effectively reduce the probability of bacterial resistance. Aldrich developed a polycaprolactone/hydroxyapatite/rifampicin mixture for the preparation of bone scaffolds. Then, daptomycin, methacrylic acid hyaluronic acid (HA), and methacrylic acylated gelatin (Gel) were mixed into hydrogels and deposited on the scaffold gap with another printing head. After the technology, six different types of drugs, such as chloramphenicol, were printed in a tablet. It can be used to treat a variety of diseases at the same time, which can not only reduce the trouble of taking a variety of drugs at one time but also control the release rate of tablets by adjusting the shape (cylindrical, circular) and internal soluble filler, which fully reflects the advantages of the technology in the preparation of combination drugs. The technical characteristics can promote the advantages of traditional Chinese medicine in antibacterial treatment. The principles of traditional Chinese medicine include monarch, minister, and assistant envoy. According to the patient's symptoms, physical fitness, age, and gender, doctors issue different prescriptions. Preparation technology can easily and quickly combine multiple traditional Chinese medicines in the same dosage form, which is convenient to take and easy to preserve. At the same time, the drug release characteristics were controlled by adjusting the printing structure, shape, type, and dosage of excipients. This kind of flexible pharmaceutical model can change drugs according to the symptoms in the process of treatment, which fully reflects the personalized characteristics of the preparation technology.

RETRACTED

As shown in Figure 3, traditional Chinese medicine and antibiotics can also be combined in the same preparation to flexibly control the proportion of drugs and print parameters to produce different efficacies. Traditional Chinese medicine can also be used to alleviate the side effects of antibiotics by adjusting the release rate. All these help to delay or prevent the occurrence of bacterial resistance and provide new strategies for the research and development of traditional Chinese medicine antibiotics. However, pharmaceutical technology still needs to rely on biological manufacturing equipment, and more equipment in line with the application characteristics of traditional Chinese medicine needs to be constantly updated and improved to jointly promote the in-depth development of this technology.

## 3. Results and Analysis

### 3.1. Antibiotic Signaling Pathway and Endocrine Resistance

As shown in Figure 4, antimicrobial peptides, Chinese herbal medicines, and other antifungal agents may be the alternative options for the treatment of Staphylococcus aureus infection in the future when the choice of effective antibiotics for the treatment of Staphylococcus aureus infection is still limited. The discovery of antibiotics is not only a great progress in the history of world medicine but also the beginning of the world drug resistance problem. Excessive use of antibiotics, or even nonstandard use, led to the emergence of bacterial resistance and formed a grim situation. The spread of drug-resistant strains is a serious public health problem because the results of conventional treatment are ineffective, which may lead to long-term infection and increase the risk of patients.

As shown in Table 1, drug resistance of Staphylococcus aureus isolated from food must be monitored for human health and food safety. It has been reported that Staphylococcus aureus has been detected from different foods at home and abroad, and the drug resistance spectrum of these pathogens has been analyzed. Dairy products are especially suitable for the growth of all kinds of bacteria, including Enterobacteriaceae, Streptococcaceae, and Bacillus, because they contain high nutrients. The total number of colonies, especially staphylococcus aureus, can exceed the standard after being contaminated by these microorganisms in dairy farms and milk processing. Staphylococcus aureus easily produces spores, and the high heat resistance of spores improves its survival rate after heat treatment. At the same time, the stronger antibiotic resistance of spores is usually considered an obstacle to the effectiveness of antibiotics and disinfectants, which may be an important reason for the higher contamination rate of Staphylococcus aureus in dairy products than other food bore pathogens.

RETRACTED

As shown in Figure 5, the use of itraconazole and voriconazole in the treatment of Aspergillus flavus infection showed a significant increase in drug resistance. There are cases that caused Trichophyton rubrum infection to reduce the sensitivity of azoles. As ketoconazole is usually used as an effective topical drug for superficial mycosis and occasionally as a reserve drug for refractory dermatophytosis, no clinical cases of ketoconazole resistance have been reported.

As shown in Figure 6, *β*-cyclodextrin inclusion achieved the local dissolution of andrographolide in the biological part, significantly improved the bioavailability of andrographolide, effectively reduced the dosage of andrographolide, and greatly enhanced the clearance efficiency of andrographolide against Staphylococcus aureus in the biological part. This kind of inclusion compound powder improves the therapeutic effect with appropriate administration mode, effective antibacterial activity, and high safety, which is a typical example of applying preparation technology to improve the antibacterial activity of traditional Chinese medicine. In addition, cyclodextrin inclusion can also reduce the irritation of the antibacterial essential oil of traditional Chinese medicine, to ensure the antibacterial effect.

As shown in Figure 7, in addition to inclusion technology and nanotechnology, microscopic image feature recognition can effectively improve the recognition accuracy of advanced preparations with the antibacterial activity of traditional Chinese medicine, especially in the preparation of wound dressing and bionic tissue. Microscopic image feature recognition is a kind of special fiber manufacturing technology, which extrudes polymer solution by a high-voltage source and atomizes under the action of static electricity.

As shown in Figure 8, antimicrobial peptides play a therapeutic role mainly by affecting the membrane and intracellular components, but with the increasing incidence of invasive candidiasis, microbial antimicrobial peptides may also produce drug resistance. Therefore, although antimicrobial peptides are expected to become an ideal drug to solve the problems of drug-resistant bacteria, virus infection, and cancer, due to their toxicity and instability, it is necessary to carry out multilevel and multiangle research on the antimicrobial mechanism and biological activity of antimicrobial peptides in the future. In conclusion, the mechanism of drug resistance of different drugs for the treatment of Staphylococcus aureus infection is quite different, and the effectiveness of some drugs and the mechanism of drug resistance formation are still unclear, so it is necessary to carry out a large number of research in this field in the future.

RETRACTED

### 3.2. Antibiotic Resistance of Cyclic Lipopeptides

As shown in Figure 9, Staphylococcus aureus's factors determine the fungal invasion pathway, infection degree, and pathogenic efficiency, and its drug resistance is also closely related to its characteristics (such as secreting special enzymes, cell membrane, cell wall, mycelium, mitochondria, and keratin adhesion resistance). Staphylococcus aureus infection of the skin, nails, and hair will accelerate the decomposition of cysteine disulfide and produce high molecular weight solid polymer structure, through the regulation of keratinase, to form and strengthen their drug resistance. The cell membrane and cell wall of Staphylococcus aureus are the most important targets of antifungal drugs. Therefore, the cell wall, cell membrane, and hyphae (phyllodes hyphae, drilling hyphae) of Staphylococcus aureus will form physical and chemical barriers during drug treatment, affecting the drug resistance of antibiotics.

As shown in Figure 10, biogenic drugs can affect the formation and adhesion of yeast germ tubes, thus reducing the toxicity of drugs to fungi. Due to its high specific surface area, adjustable nanoscale and porosity, and sustained drug release, the dressing can effectively improve the antibacterial ability of BER. The dressing prepared by using the microscopic image feature recognition technology can not only be used for antibacterial but also prevent the penetration of exogenous bacteria. It can be used as an ideal production method of antibacterial dressing and has broad prospects in improving the antibacterial effect of drugs and treating bacterially infected wounds. In addition to being used as a wound antibacterial dressing, microscopic image feature recognition technology also has advantages in the synthesis of artificial periosteum with antibacterial activity.

As shown in Figure 11, antibiotic resistance inhibition can precisely mimic the natural periosteal structure and bone formation function by reasonably adjusting the polymer fiber structure and effectively improve the antibacterial effect of materials combined with antibacterial drugs, giving play to the antibacterial advantages of traditional Chinese medicine. This kind of microscope image feature recognition manufacturing technology opens up a new scene and new form of antibacterial application of traditional Chinese medicine, which is worthy of further exploration. In addition to these manufacturing technologies, there are also some physical and chemical methods to improve the antibacterial activity of traditional Chinese medicine. Modification techniques such as physical crosslinking, electrostatic adsorption, chemical crosslinking, and conjugation synthesis can also improve the antibacterial efficacy of traditional Chinese medicine to a certain extent. However, these methods still have some defects, such as narrow application scope, high cost, and limited practical application.

RETRACTED

The advantage of the AMR (activity metabolic rate) index in the antibacterial aspect is shown in Figure 12. Most of the strains carried only one per gene, including three strains carrying Qnrb, nine strains carrying cars, and one strain carrying Qnrd. The per gene form of four strains was in Oqxb.

It is an effective solution to improve the antibacterial activity of traditional Chinese medicine through preparation technology. As shown in Figure 13, inclusion technology, nanotechnology, and microscopic image feature recognition technology have good application effects in improving the antibacterial activity of a single prescription of traditional Chinese medicine. However, the antibacterial activity of traditional Chinese medicine compound preparations or preparations combined with antibiotics is better. Therefore, how to improve the preparation technology to obtain more stable and efficient traditional Chinese medicine compound preparations or preparations combined with Chinese and Western medicine is a key problem for the preparation field workers. Based on this, this paper focuses on a drug preparation technology, which has outstanding advantages in the preparation of personalized antibacterial agents and combination antibacterial agents and can provide ideas and references for the preparation of compound Chinese medicine antibacterial agents and a combination of Chinese and Western medicines. At present, there is no report on the improvement of the antibacterial activity of traditional Chinese medicine by preparation technology.

## 4. Discussion

In recent years, the drug resistance of Staphylococcus aureus to terbinafine has also increased year by year. For example, in patients with congenital ichthyosis or chronic tinea corporis, after increasing and continuous exposure to terbinafine, drug resistance has been obtained. In this paper, the characteristics and advantages of these preparation technologies are introduced from the two aspects of single-prescription antibacterial traditional Chinese medicine preparation technology and combined antibacterial drug preparation technology. The application of these two kinds of preparation technology in improving the antibacterial activity of drugs is reported, and their shortcomings are compared and analyzed. Our research group has been committed to the rapid detection of control bacteria in traditional Chinese medicine products and systematically summarized the technology in the early stage, which laid a scientific foundation for the writing of this paper. A large number of studies have shown that Trichophyton interphalangeal and Trichophyton rubrum isolated from patients with onychomycosis, tinea pedis, and tinea corporis is highly resistant to terbinafine. In the study of drug resistance of pathogenic dermatophytes to terbinafine, 47% of patients showed drug resistance to terbinafine. However, Trichophyton rubrum isolated from patients with tinea pedis and onychomycosis in Switzerland had only 1% drug resistance to terbinafine, while Trichophyton mentagrophytes had 30%-70% drug resistance, which suggested that the resistance of fungal infection to allylamine might be related to individual differences and the types of Staphylococcus aureus infection.

RETRACTED

At present, there are few studies on the mechanism of drug resistance of nano-CuO. Because nano-CuO can act on multiple targets of Staphylococcus aureus, affect mitochondrial respiratory chain to produce reactive oxygen species, regulate calcium homeostasis, and so on, this special mechanism can effectively prevent Staphylococcus aureus from producing drug resistance. However, some specific groups of Staphylococcus aureus are resistant to nano-CuO. For example, Candida albicans strains with gene mutation have high resistance to amphotericin B. In addition, a study in Kuwait found that 10% of Aspergillus flavus strains isolated from clinical and environmental samples showed resistance to amphotericin. Therefore, the resistance of Staphylococcus aureus to nano-CuO is related to the species of fungi. This paper reviews the application of different preparation technologies in improving and enhancing the antibacterial activity of traditional Chinese medicine from the perspective of preparation, including inclusion technology, nanotechnology, microscope image feature recognition technology, image recognition technology, and some other technologies. The principles of these technologies are different, so are their advantages and disadvantages. Inclusion technology, nanotechnology, and microscopic image feature recognition technology have a certain effect in improving the antibacterial activity of single-prescription or single-component traditional Chinese medicine preparations, while technology has the most obvious advantage in improving the antibacterial activity of traditional Chinese medicine compound preparations. It can freely adjust the printing structure and shape to meet different drug needs and can flexibly select drugs or excipients to achieve different drug release activities; it has great flexibility and combination in the preparation of compound antibacterial drugs. The systematic introduction of different preparation technologies in improving the antibacterial activity of traditional Chinese medicine has not been reported.

RETRACTED

Microscope image technology is a new drug preparation technology, which is applied more and more in the field of medicine and pharmacy. At present, there are many types of the molding process, which has a wide range of adaptability and strong flexibility. Through the technology, the printing parameters of drugs can be flexibly modified to print personalized antibacterial drugs, to achieve a variety of drug release activities. In addition, multiple drugs can be combined in the same dosage form to realize the synergistic effect of combined drugs. These outstanding advantages can be used to improve and enhance the antibacterial properties of compound Chinese medicine, which makes up for the shortcomings of conventional preparation technology.

As an important host of Salmonella, the threat of human infection caused by pets should be paid more attention to. Especially in recent ten years, the rapid expansion of the number of pets in China and the increase of drug dosage caused by the aging of pets lead to the increase of drug-resistant strains in the body, which makes the threat of drug-resistant Salmonella to public health not ignored. The carrying rate of Salmonella in pets in the Beibei District of Chongqing was about 4%, which was lower than that in Urumqi and Xuzhou, but similar to that in Hefei. The antimicrobial resistance rate of Salmonella isolated in Beibei District was lower than that in other areas, but the proportion of multidrug-resistant strains was higher, 10 multidrug-resistant strains accounted for 82.93% of the total number of isolated strains, and there were five or six drug-resistant strains. Salmonella is a kind of intestinal bacteria in pets. When people have close contact with pets, they may be infected with Salmonella carried by pets. When people's immunity is decreased or immune function is not perfect, Salmonella from pets may cause disease. If it is drug-resistant bacteria, it will increase the treatment time and cost, and even there is no drug available. Therefore, to strengthen the drug resistance monitoring of Salmonella from pets and clarify the main drug resistance genes of Salmonella from pets can provide a reference for drug use of Salmonella from pets and provide early warning for human infection with Salmonella from pets. In this study, an epidemiological investigation was conducted on Salmonella from pets in Beibei District of Chongqing City, and the susceptibility of the isolated strains to some antibiotics was determined *β*-extended-spectrum *Β*- to provide a reference for the drug use of pet Salmonella and human infected with pet Salmonella in Beibei District.

RETRACTED

In summary, medical image feature recognition technology can improve the antibacterial properties of Chinese medicine to a certain extent, which is beneficial to improving the current status of clinical antibacterial treatment. However, there are still some problems in the application of these technologies, such as the low encapsulation efficiency of inclusion technology, metal nanoparticles easily produce cytotoxicity in vivo, and the degree of nano-self-assembly is low.

## 5. Conclusions

Traditional medicine manufacturing technology is often limited to improving or enhancing the antibacterial activity of one or a class of Chinese medicines. In other words, these preparation technologies are relatively effective in improving the antibacterial activity of a single Chinese medicine or a single active ingredient, but the preparation of multiple antibacterial compatibilities of Chinese medicines is often limited. In the study of antibiotic resistance based on intelligent medical imaging, nano-CuO also showed a certain degree of cyclic lipopeptide resistance in clinical applications. For example, with the widespread use of echinocandin, more and more cases of Staphylococcus aureus resistance to echinocandin have been reported. After the use of echinocandin drugs, the pathogens of Staphylococcus aureus will adapt to the drugs over time. For example, Candida and Aspergillus are significantly resistant to echinocandin drugs after exposure. In addition, genetic mutations may also cause fungi to mutate during reproduction and acquire inherent resistance. In the future, we will develop more new preparations suitable for exerting the antibacterial activity of compound Chinese medicines and effectively improve the antibacterial effect of Chinese medicines. This article will closely combine the technical characteristics of the preparations and the advantages of the compatibility of Chinese medicines and use advanced medical imaging systems under the guidance of Chinese medicine theories to prepare more flexible and effective Chinese medicine antibacterial compounds. The antibacterial agents proposed in this article provide new ideas and strategies for solving the problem of bacterial resistance.

## Figures and Tables

**Figure 1:** Antibiotic drug release kinetics and drug resistance.

**Figure 2:** Time effect and therapeutic effect of drugs.

RETRACTED

**Figure 3:** Adjust the release rate of the frame of FIG to alleviate the side effects.

**Figure 4:** Line graph with limited options for antibiotics.

**Figure 5:** Sensitivity of Trichophyton infection to azole drugs.

**Figure 6:** Staphylococcus aureus removal efficiency.

**Figure 7:** Antibacterial activity of plant essential oils.

**Figure 8:** The therapeutic effect of thin membrane and intracellular components.

**Figure 9:** Pass rate of different concentrations of Staphylococcus aureus.

**Figure 10:** Yeast bud tube formation and adhesion.

**Figure 11:** Precisely bionic natural periosteal structure.

**Figure 12:** AMR compound antibacterial Chinese medicine preparation technology.

**Figure 13:** AMR compound preparation or Western medicine combination preparation.

**Table 1:** Staphylococcus aureus resistance.

Item	Research source	Escherichia coli	Resistance	Rate	Variability
Acinetobacter baumannii	5.42	6.07	7.73	5.84	7.88
Antibacterial drugs	4.03	6.29	7.64	6.63	6.57
Klebsiella pneumoniae	2.3	5.37	7.83	7.57	6.48
Clinical distribution	2.56	3.93	6.15	8.29	7.09
Sensitivity	2.72	3.95	4.88	8.57	5.38

## Data Availability

The data that support the findings of this study are available from the corresponding author upon reasonable request.
